# Medical Data Acquisition and Internet of Things Technology-Based Cerebral Stroke Disease Prevention and Rehabilitation Nursing Mobile Medical Management System

**DOI:** 10.1155/2022/4646454

**Published:** 2022-01-28

**Authors:** Yunna Song, Wenjing Zhang, Qingjiang Li, Wenhui Ma

**Affiliations:** ^1^Mathematics Teaching and Research Section, Qiqihar Medical University, Qiqihar, 161000, China; ^2^Teaching and Research Section of Computer Science, Qiqihar Medical University, Qiqihar 161000, China; ^3^Computer Experimental Teaching Center, Qiqihar Medical University, Qiqihar 161000, China

## Abstract

This research was aimed at exploring the application value of a mobile medical management system based on Internet of Things technology and medical data collection in stroke disease prevention and rehabilitation nursing. In this study, on the basis of radio frequency identification (RFID) technology, the signals collected by the sensor were filtered by the optimized median filtering algorithm, and a rehabilitation nursing evaluation model was established based on the backpropagation (BP) neural network. The performance of the medical management system was verified in 32 rehabilitation patients with hemiplegia after stroke and 6 healthy medical staff in the rehabilitation medical center of the hospital. The results showed that the mean square error (MSE) and peak signal-to-noise ratio (PSNR) of the median filtering algorithm after optimization were significantly higher than those before optimization (*P* < 0.05). When the number of neurons was 23, the prediction accuracy of the test set reached a maximum of 89.83%. Using traingda as the training function, the model had the lowest training time and root mean squared error (RMSE) value of 2.5 s and 0.29, respectively, which were significantly lower than the traingd and traingdm functions (*P* < 0.01). The error percentage and RMSE of the model reached a minimum of 7.56% and 0.25, respectively, when the transfer functions of both the hidden and input layers were tansig. The prediction accuracy in stages III~VI was 90.63%. It indicated that the mobile medical management system established based on Internet of Things technology and medical data collection has certain application value for the prevention and rehabilitation nursing of stroke patients, which provides a new idea for the diagnosis, treatment, and rehabilitation of stroke patients.

## 1. Introduction

Cerebral stroke is a common acute cerebrovascular disease, and its clinical manifestations are local neurological deficits [1]. Cerebral stroke is the second largest cause of death and the first cause of disability worldwide, with high morbidity, high disability rate, high mortality, and high recurrence rate [2]. In recent years, with the intensification of population aging in China, the incidence of cerebral stroke patients increased significantly. According to statistics, there are about 2.46 million new cases of cerebral stroke each year in China, of which about 75% of the patients cannot live independently due to disability, and more than 40% are severely disabled [3]. Due to the characteristics of cerebral stroke disease, its treatment activities have strong real-time performance and are often accompanied by complications such as dysfunction after rehabilitation [4]. The current research results show that early rehabilitation nursing can promote the cerebral cortex reorganization of patients with cerebral nerve injury and help to restore the body [5]. Due to the influence of medical conditions and hospitalization expenses, patients cannot be treated in hospitals for a long time, and the number and quality of nursing staff in community rehabilitation centers cannot meet the needs of nursing for cerebral stroke patients [6].

In recent years, with the continuous development of computer technology and Internet of Things technology, mobile medical and health service systems are gradually applied to the prevention, diagnosis, treatment, and nursing of diseases and have become a new type of medical and health care model [7]. The Internet of Things is an intelligent network system that realizes information exchange and communication through network connection of information sensing devices such as radio frequency identification (RFID) technology, infrared sensing, and global positioning system [8]. The medical mobile APP based on Internet of Things technology realized the detection and management of patients' body temperature, blood pressure, blood glucose, and heart rate. It can communicate with doctors in real time through remote medical system and improve the accuracy of disease diagnosis and treatment and the quality of medical service [9, 10]. In addition, the rise of big data also provides favorable conditions for the rapid development of medical informatization. Medical data ensure the continuity of individual medical treatment, and at the same time, the health status of patients can be analyzed and predicted based on the data of patients' health information [11]. While the medical and health service platform based on Internet of Things technology provides convenience for patient diagnosis and treatment, it also has the disadvantages of lack of sharing of health information, lack of continuous monitoring and management of health physiological parameters, and inability to meet multilevel health needs. The prevention and rehabilitation tracking of cerebral stroke patients can timely evaluate the rehabilitation of patients and prevent the recurrence of the disease. At present, most medical institutions focus on the diagnosis and treatment of cerebral stroke patients [12], ignoring the prevention and rehabilitation tracking of cerebral stroke patients.

In summary, there are few studies on the mobile management system for disease prediction and rehabilitation nursing tracking of cerebral stroke patients. Based on the mobile medical monitoring system and combined with RFID technology, this study studies the tracking and management of the prevention and rehabilitation process of cerebral stroke patients, so as to establish a mobile medical management system for cerebral stroke disease prevention and rehabilitation nursing, and improve the timeliness and efficiency of cerebral stroke disease diagnosis.

## 2. Materials and Methods

### 2.1. Design of Mobile Medical System Based on Internet of Things

The remote mobile medical monitoring system for cerebral stroke patients based on Internet of Things is mainly composed of three layers: physiological parameter acquisition node (data access layer), business logic layer, and intelligent mobile Android terminal layer. The data access layer mainly identifies and transmits the basic clinical data of patients through PDA equipment according to the RFID tag carried by patients, including the hospital information system (HIS) such as patients' physiological characteristics and signs. The business logic layer mainly processes and analyzes the data through mobile hospital information system (MobHIS) and network platform. The intelligent mobile Android terminal layer receives, processes, and displays patient disease information. The framework of the mobile medical system based on Internet of Things in this study is illustrated in Figure 1.

In this study, the wireless intrusion detection system (WIDS) and wireless network controller (WNC) are mainly used as the medical dedicated wireless network system. WIDS realizes that multiple networks cover a target area at the same time through multifrequency combination and can realize the linear expansion of the wireless network capacity [13]. WNC can ensure the security and stability of the wireless network system [14].

### 2.2. Structure Design of Cerebral Stroke Rehabilitation Mobile Monitoring System

In this study, a mobile monitoring system model of human-computer interaction is established by combining remote communication technology, computer intelligence technology, and rehabilitation nursing methods. Cerebral stroke prevention and rehabilitation mobile monitoring system is mainly composed of two modules: patient clinical data acquisition and remote cerebral stroke rehabilitation nursing. The clinical data acquisition mainly obtains the patient's identification (ID) and clinical information by scanning RFID wristband tags and acceleration sensors; transmits the data to the rehabilitation nursing database through the Internet; preprocesses and identifies the data through the rehabilitation nursing system, such as denoising and normalization; and finally obtains the rehabilitation nursing results. The doctor shall timely feedback the recovery status of patients according to the results of the rehabilitation nursing system. The structure diagram of the cerebral stroke rehabilitation nursing mobile monitoring system is shown in Figure 2.

### 2.3. Data Acquisition and Processing of Cerebral Stroke Rehabilitation Mobile Monitoring System

The data related to rehabilitation training are collected by binding three-dimensional acceleration sensors to the patient's forearm and upper arm. The collected data are transmitted to the wireless data receiver through the built-in Zigbee wireless transmission module and uploaded to the client software system. It is assumed that the accelerations of the acceleration sensor in three directions are *A*_*x*_, *A*_*y*_, *A*_*z*_, and the calculation method of sensor roll angle *α* and pitch angle *β* is as follows.

(1) $$\begin{array}{c} \alpha =\arctan\left(\frac{A_{x}}{A_{z}}\right),\\ \beta =\arctan\left(\frac{A_{\text{y}}}{A_{z}}\right). \end{array}$$

Signals are often disturbed by random noise or Gaussian noise in the process of generation and transmission. The commonly used signal filtering methods include linear filtering and nonlinear filtering [15]. Linear filtering has better denoising effect on Gaussian white noise but worse on impulse noise [16]. The median filtering method in nonlinear filtering has good suppression ability for a narrow pulse signal, but its filtering effect on Gaussian white noise needs to be further optimized [17]. For the median filter with filter window side length *n*, it can be expressed as follows.

(2) $$\begin{array}{c} y_{i}=\text{med}\left(f_{i-n},f_{i-n+1},\cdots ,f_{i+n}\right). \end{array}$$

med represents the extraction median function and *f*_*i*−*n*_, *f*_*i*−*n*+1_, ⋯, *f*_*i*+*n*_ represents the result sequence of one-dimensional odd window. The two-dimensional median filter slides in the image in order, and its calculation method is as follows.

(3) $$\begin{array}{c} y_{i\text{j}}=\text{med}\left\{x_{ij}\right\}. \end{array}$$

*x*_*ij*_ is the pixel value of the input area for the window, and *y*_*i*j_ represents the intermediate value after sorting the pixel values in the window area. The median filter input signals are Gaussian distributed, and the approximate noise variance can be expressed as follows.

(4) $$\begin{array}{c} \chi_{\text{med}}^{2}=\frac{1}{4{mg}^{2}\left(n^{\prime }\right)}=\frac{\chi_{i}^{2}}{n+\pi /2-1}\times \frac{\pi }{2}. \end{array}$$

*n*′ is the noise mean, *χ*_*i*_^2^ represents the input noise variance, *n* represents the filter window length, and *g*^2^(*n*′) represents the noise density function.

The output noise distribution of the median filter has a certain correlation with the input noise model and the probability density distribution [18]. The frequency response calculation method of median filtering system can be expressed as follows.

(5) $$\begin{array}{c} A=\left|\frac{C}{F}\right|. \end{array}$$

*A* represents the frequency response of median filter system, and *C* and *F* represent the spectrum of input signal and output signal.

For the check noise processing in the data, pixelmedianfiler(*N*, *i*, *j*, *A*) function is introduced to optimize it. It is assumed that the pixel position before filtering is (*i*, *j*); the row vector of the filtered pixel position template matrix can be expressed as follows:

(6) $$\begin{array}{c} \text{pixelset}=\text{adipixel}\left(N,i,j,A\right). \end{array}$$

Due to the limited motor function of cerebral stroke rehabilitation patients, most patients cannot accurately complete the prescribed rehabilitation nursing actions. The obtained data need to further extract the physical characteristics of the signal. The physical characteristics of the signal mainly include the root mean square (RMS), variance, and energy characteristics. The calculation method is as follows.

(7) $$\begin{array}{c} \text{RMS}={\left(\frac{1}{N}\overset{N}{\underset{\text{i}=1}{\sum }}x_{i}^{2}\right)}^{1/2},\\ \text{Var}=\frac{1}{N-1}\overset{N}{\underset{\text{i}=1}{\sum }}{\left(x_{i}-\delta \right)}^{2},\\ \text{En}=\overset{N}{\underset{\text{i}=1}{\sum }}\left|B_{i}\right|. \end{array}$$

RMS is the root mean square, Var is the variance, En is the energy characteristic, *N* is the sequence length, *δ* is the mean, and *B*_*i*_ is the signal Fourier transform amplitude.

Mean square error (MSE), root mean square error (RMSE), and peak signal-to-noise ratio (PSNR) were used to evaluate the filtered data. The MSE, RMSE, and PSNR were calculated as follows.

(8) $$\begin{array}{c} \text{MSE}=\frac{1}{m}\overset{m}{\underset{i=1}{\sum }}\overset{m}{\underset{j=1}{\sum }}{\left[X\left(i,j\right)-Y\left(i,j\right)\right]}^{2},\\ \text{RMSE}=\sqrt{\frac{1}{m}\overset{m}{\underset{i=1}{\sum }}\overset{m}{\underset{j=1}{\sum }}{\left[X\left(i,j\right)-Y\left(i,j\right)\right]}^{2}},\\ \text{PSNR}\left(X,Y\right)=10\log_{10}\left(\frac{L^{2}}{\text{MSE}\left(X,Y\right)}\right). \end{array}$$

(i, *j*) is the pixel position, *m* is the number of measurements, *X* is the measured value, *Y* is the true value, *L* is the peak signal, and MSE(*X*, *Y*) is the MSE of the image.

### 2.4. Establishment of Cerebral Stroke Rehabilitation Nursing Evaluation Model

The back propagation (BP) neural network learns a certain number of sample pairs. After the hidden layer and output layer are calculated, the predicted values of each neuron output in the output layer are calculated. Through the back propagation error, the error between the network, output, and expected output is gradually reduced [19]. For the sample pair (*X*, *Y*), the calculation method of the network weight matrix *W*_1_ between the input layer and the hidden layer neurons and the network weight matrix *W*_2_ between the hidden layer and the output layer neurons are as follows.

(9) $$\begin{array}{c} W_{1}=\left[\begin{array}{ccccc} w_{11}^{1} & \; & w_{12}^{1} & \cdots & w_{1m}^{1}\\ w_{21}^{1} & \; & w_{22}^{1} & \cdots & w_{2m}^{1}\\ \; & \vdots & \; & \cdots & \vdots \\ w_{l1}^{1} & \; & w_{l2}^{1} & \cdots & w_{lm}^{1} \end{array}\right],\left[\begin{array}{ccccc} w_{11}^{2} & \; & w_{12}^{2} & \cdots & w_{1l}^{2}\\ w_{21}^{2} & \; & w_{22}^{2} & \cdots & w_{2l}^{2}\\ \; & \vdots & \; & \cdots & \vdots \\ w_{n1}^{2} & \; & w_{n2}^{2} & \cdots & w_{nl}^{2} \end{array}\right]. \end{array}$$

The threshold *σ*_1_ of the hidden layer neuron and the threshold *σ*_2_ of the output layer neuron can be expressed as follows.

(10) $$\begin{array}{c} \sigma_{1}=\left[\sigma_{1}^{1},\sigma_{2}^{1},\cdots ,\sigma_{l}^{1}\right],\sigma_{2}=\left[\sigma_{1}^{2},\sigma_{2}^{2},\cdots ,\sigma_{n}^{2}\right]. \end{array}$$

The output *O*_*j*_ of the hidden layer neuron and the output *Z*_*k*_ of the output layer neuron are expressed as follows.

(11) $$\begin{array}{c} O_{j}=f\left(\overset{m}{\underset{i=1}{\sum }}w_{ij}^{l}x_{i}-\sigma_{l}^{i}\right)=f\left({\text{net}}_{j}\right),\;j=1,2,\cdots ,l,\\ Z_{k}=g\left(w_{kj}^{2}O_{j}-\sigma_{k}^{2}\right)=g\left({\text{net}}_{k}\right),\;k=1,2,\cdots ,n. \end{array}$$

*f*() represents the transfer function of the hidden layer, and *g*() is the transfer function of the output layer.

The error between network output and expected output of the BP neural network can be expressed as follows.

(12) $$\begin{array}{c} E=\frac{1}{2}\overset{n}{\underset{\text{k}=1}{\sum }}\left(y_{k}-z_{k}\right)=\frac{1}{2}\overset{n}{\underset{\text{k}=1}{\sum }}{\left[y_{k}-g\left(\overset{l}{\underset{j=1}{\sum }}w_{kj}^{2}O_{j}-\sigma_{k}^{2}\right)\right]}^{2}. \end{array}$$

The number of hidden layer neurons has a significant impact on the performance of the BP neural network. The number of hidden layer neurons can be calculated by empirical equation.

(13) $$\begin{array}{c} n=\frac{a+b}{2}+c. \end{array}$$

*a* and *b* are the number of neurons in the input layer and the output layer, respectively, and *c* is the constants within 10.

### 2.5. Database Design and Test Environment of Cerebral Stroke Rehabilitation Mobile Monitoring System

The database and its application system are the core and foundation of the database design of the mobile monitoring system. The design of the database needs to meet the principles of integrity, small number, small number of fields, and high efficiency [20]. Storage and access methods are the main physical structure of the database [21]. The physical structure of the database needs to meet the minimum storage space and improve the effective access efficiency of the database [22]. The physical object of this database involves the patient entity and rehabilitation data entity, and the main physical structure includes the patient information table, rehabilitation data table, rehabilitation exercise prescription table, and rehabilitation data information table. The specific information in the database is shown in Tables 1–4.

The test system running the platform environment is as follows: computer operating system Windows 10 flagship version 64-bit operating system, server-side scripting language PHP 5.3.5, relational database management system MySQL 5.5.8, and web server software Apache 2.2.17. The development environment is as follows: project development compiler EclipsePHP studio3, data management library PhpMyAdmin3.39, and Javascript and Ajax are used as code programming tools.

### 2.6. Verification of Cerebral Stroke Rehabilitation Mobile Monitoring System

The rehabilitation of cerebral stroke patients was evaluated by the Brunnstrom staging method. According to the results of Wang et al. [23], the motor function recovery of patients was divided into 6 grades: stage I: no muscle contraction, stage II: combined reaction occurred, stage III: collaborative movement was launched at will, stage IV: separation movement occurred, phase V: relatively independent comovement occurred, and stage VI: near normal or basically normal.

32 hemiplegic rehabilitation patients after cerebral stroke and 6 healthy medical staff from the hospital from December 2019 to March 2021 were selected as the research objects. The motion quality was evaluated according to the acceleration physical characteristics collected in the process of the rehabilitation nursing exercise. Most of the cerebral stroke patients were in Brunnstrom stages II-V, and the 6 medical staff were in the stage VI rehabilitation group. Patients with severe cognitive or communication disorders were excluded. 75% of the data were randomly selected from Brunnstrom cerebral stroke patients at different stages as the training set and the remaining 25% as the test set.

The rehabilitation nursing method refers to the method of Ikbali et al. [24] to carry out the standard movement training of “patient's hand touching shoulder,” and it is modified accordingly. The patient's upper limb rehabilitation training is mainly completed according to the motion guidance map. At the beginning of the training, the user can choose the guidance map freely according to preferences and the upper limb use habits. The action of each cycle takes 10 seconds as the sampling cycle.

### 2.7. Statistical Methods

The test data were processed by SPSS19.0 statistical software. The measurement data were expressed by mean ± standard deviation ($\overset{¯}{\text{x}}\pm \text{s}$), and *t*-test was used. The counting data was expressed by percentage (%). *P* < 0.05 indicated that the difference was statistically significant.

## 3. Results and Analysis

### 3.1. Comparison of Indicators before and after Filter Optimization

The signal processing results before and after the optimization of the median filtering algorithm are compared and analyzed. With the increase of noise intensity, the mean square error (MSE) of the signal showed a significant upward trend. When the noise intensity was 5%, 10%, 20%, 40%, and 60%, the MSE values of the optimized median filtering algorithm were 54.17 ± 4.52, 103.52 ± 8.63, 215.42 ± 17.95, 1302.17 ± 108.51, and 4865.22 ± 455.26, respectively, and the MSE values of the median filtering algorithm before optimization were 2.17 ± 0.34, 15.41 ± 1.48, 21.52 ± 1.99, 52.42 ± 4.87, and 116.92 ± 8.63, respectively. At different noise intensities, the MSE values of the median filtering algorithm after optimization were significantly inferior than those before optimization, and there was a highly significant difference between the two (*P* < 0.001) (Figure 3). The peak signal-to-noise ratio (PSNR) value of the optimized median filtering algorithm was significantly higher than that before optimization (*P* < 0.05) (Figure 4). It suggested that the median filtering algorithm has better denoising and smoothing performance for the image after optimization, which may be due to the introduction of pixelmedianfiler(*N*, *i*, *j*, *A*) function in the optimization algorithm, which can filter all noise points at one time, but also well preserve the image details and enhance the noise reduction effect of the median filtering algorithm.

### 3.2. Signal Filtering Processing Result Analysis

The signals recorded by the upper arm sensor during the rehabilitation nursing training of patients were analyzed. Before filtering, the signals in different directions contained obvious linear noise and calibration noise. The optimized median filter was used to filter the signals. The interference waveforms in the signal curves of the upper arm sensors in different directions of *X*, *Y*, and *Z* axes were significantly reduced (Figure 5).

### 3.3. Determination of Neuron Number in Cerebral Stroke Rehabilitation Nursing Evaluation Model

The root mean square error (RMSE) values of the model under different numbers of neurons in the hidden layer were analyzed (Figure 6). With the increase of the number of neurons, the RMSE value of the model showed a trend of increasing and then decreasing. When the number of neurons was greater than 23, the RMSE value of the model tended to be stable and the change was small. Under different numbers of neurons, the prediction accuracy of the training set and the test set was different. When the number of neurons was 23, the prediction accuracy of the test set reached the maximum value of 89.83%, the prediction accuracy of the test set decreased rapidly, and the prediction accuracy of the training set showed a stable state (Figure 7). Therefore, the number of neurons in the hidden layer was selected as 23 in this study.

### 3.4. Function Selection of Cerebral Stroke Rehabilitation Nursing Evaluation Model

At present, the training functions for the BP neural network algorithm mainly include the traingd function of the gradient descent algorithm, traingdm function of the momentum backpropagation gradient descent, and traingda function of the dynamic adaptive learning rate [25]. In this study, the training time and RMSE values under three different training functions are compared (Figure 8). Traingda was used as the training function, the training time and RMSE value of the model were the lowest, which were 2.5 s and 0.29, respectively. The training time and RMSE value of traingda were significantly lower than those of traingd and traingdm functions (*P* < 0.01). The training steps of the traingda training function were significantly different from those of traingd and traingdm functions (*P* < 0.001), so traingda was selected as the training function.

The transfer function has a significant influence on the prediction accuracy of the neural network. At present, the commonly used node transfer functions are logsig, tansig, and purelin functions [26]. The error percentage and RMSE values under different transfer functions in the hidden layer and the input layer are compared (Figure 9). When the transfer in the hidden layer and the input layer is tansig, the error percentage and RMSE values of the model are the minimum, which are 7.56% and 0.25, respectively.

### 3.5. Result Analysis of Cerebral Stroke Rehabilitation Mobile Monitoring System

The Brunnstrom staging results of the subjects included in the study were compared with the prediction results of the mobile monitoring system (Figure 10). In 32 samples, the prediction results of stages I and II were completely consistent with the clinical staging results. There were 3 samples (9.37%) with difference between normal prediction results and clinical stage results in stages III-VI, and the prediction accuracy was 90.63%. With the increase of the stage grade, the error rate of prediction results increases. It is analyzed that the reason may be caused by the unstable rehabilitation status of the research object and the lack of test data.

## 4. Conclusion

In this study, a mobile medical management system for stroke prevention and rehabilitation care was established based on Internet of Things technology and medical data collection, and the results revealed that the system was feasible. However, there are still some shortcomings: the number of cases is small and the amount of collected data is insufficient, so the number of cases will be increased in the future work to further evaluate the rehabilitation nursing model and management system. In conclusion, the rehabilitation nursing mobile medical management system established based on Internet of Things technology and medical data collection has certain application value for the prevention and rehabilitation nursing of stroke patients, which provides a new idea for the diagnosis, treatment, and rehabilitation of stroke patients.

## Figures and Tables

**Figure 1:** Framework of mobile medical system based on Internet of Things.

**Figure 2:** Structure diagram of cerebral stroke rehabilitation nursing mobile monitoring system.

**Figure 3:** Comparison of MSE values of median filtering algorithm under different noise intensities. (∗∗ represents a significant difference compared to preoptimization, *P* < 0.001.)

**Figure 4:** Comparison of PSNR values of median filtering algorithm under different noise intensities. (∗∗ represents that there is significant difference compared to preoptimization, *P* < 0.05.)

**Figure 5:** Motion signal curves in different directions: (a) upper arm sensor *X*-axis; (b) upper arm sensor *Y*-axis; (c) upper arm sensor *Z*-axis.

**Figure 6:** RMSE value distribution of the model under different numbers of neurons.

**Figure 7:** Prediction accuracy of test set and training set under different numbers of neurons.

**Figure 8:** Indicator comparison of different training functions: (a) training time and RMSE value; (b) training steps. (∗∗ indicates a significant difference compared with traingda, *P* < 0.01. ∗∗∗ indicates a highly significant difference compared with traingda, *P* < 0.001.).

**Figure 9:** Performance comparison of transfer function between hidden layer and output layer.

**Figure 10:** Distribution of predicted staging and clinical staging.

**Table 1:** Basic information of patients.

Field name	Data type	Whether to type	Length	Note
ID code	Int	Yes	20	Not null
Name	Tinyint	No	5	Not null
Gender	Varchar	No	2	Not null
Age	Datetime	No	0	Not null
Marital status	Varchar	No	10	Null
Occupation	Varchar	No	10	Not null
Educational level	Varchar	No	10	Not null

**Table 2:** Patient rehabilitation data.

Field name	Data type	Whether to type	Length	Note
ID code	Int	Yes	20	Not null
Past medical history	Varchar	No	400	Not null
Marriage history	Datetime	No	50	Not null
Diagnostic time	Year	No	4	Not null
Rehabilitation assessment	Varchar	No	400	Not null
Clinical diagnosis	Varchar	No	200	Not null
Rehabilitation goal	Int	No	120	Null
Rehabilitation plan	Varchar	No	40	Null

**Table 3:** Patient rehabilitation exercise prescription.

Field name	Data type	Whether to type	Length	Note
ID code	Int	No	20	Not null
Doctor ID	Int	No	20	Not null
Prescription formulation time	Datetime	Yes	0	Not null
Prescription content	Varchar	No	500	Not null

**Table 4:** Patient rehabilitation data statistics.

Field name	Data type	Whether to type	Length	Note
ID code	Int	Yes	20	Not null
Data type	Int	No	11	Not null
Data name	Varchar	No	50	Not null
Data content	Mediumblob	No	0	Not null
Score	Int	No	5	Not null
Stage results	Varchar	No	5	Not null

## Data Availability

The data used to support the findings of this study are available from the corresponding author upon request.
